The article "Molecular Mechanism of Dayuan Decoction in the Treatment of Fever Based on Network Pharmacology" was published in 2022. Journal: Comput Math Methods Med.

# Molecular Mechanism of Dayuan Decoction in the Treatment of Fever Based on Network Pharmacology

**DOI:** 10.1155/2022/7422383

**Published:** 2022-03-25

**Authors:** Tielin Ye

**Affiliations:** Shandong Second Provincial General Hospital, Jinan 250022, China

## Abstract

**Objective:**

To study the molecular targets and mechanisms of Dayuan Decoction in the treatment of fever.

**Methods:**

The traditional Chinese medicine system pharmacological database and analysis platform (TCMSP) was used to search for the main active components and action targets of Dayuan Decoction. The GeneCards database was used to retrieve fever-related gene targets. The common gene targets were obtained by selecting the intersection of the action targets of the main active components of Dayuan Decoction and the fever-related gene targets using a Wayne diagram. Cytoscape 3.7.2 software was used to construct the drug active component action target network diagram. The protein-protein interaction PPI network of coacting targets was constructed using the STRING database. David data were used for Gene Ontology (GO) and the Kyoto Encyclopedia of Genes and Genomes (KEGG) pathway enrichment analyses of common gene targets.

**Results:**

A total of 89 main active components and 832 acting gene targets of Dayuan Decoction were screened, of which 50 were common gene targets of Dayuan Decoction and fever, including apoptosis regulatory factor Bel (BCL2L1), interleukin 6 (IL-6), interleukin 10 (IL-10), and tumor necrosis protein 53 (TP53). A total of 47 GO and 59 KEGG enrichment entries were obtained using GO and KEGG enrichment analyses, involving the cancer pathway, hypoxia-inducible factor 1 (HIF-1) signaling pathway, and mitogen-activated protein kinase (MAPK) signaling pathway.

**Conclusion:**

Dayuan Decoction has multitarget regulation characteristics and a multifaceted role in the treatment of fever.

## 1. Introduction

The heat generation and dissipation processes of the human body maintain a dynamic equilibrium under the supervision of the temperature regulation center [1]. When the body is subjected to a heat source or malfunction of the temperature center, the heat generation process increases, but the heat dissipation process cannot increase or decrease in proportion. Fever is a body temperature of 37.3°C or higher. Infectious fever (fever produced by the invasion of numerous pathogens, such as bacteria (*Mycoplasma pneumoniae*, *Rickettsia* sp., and spirochetes), fungi, and parasites), and noninfectious fever are both prevalent. The typical normal human body temperature is between 36 and 37°C (armpit). Low heat is 37.3–38°C, medium heat is 38.1–39°C, high heat is 39.1–41°C, and ultrahigh heat is >41°C.

The article "Molecular Mechanism of Dayuan Decoction in the Treatment of Fever Based on Network Pharmacology" was published in 2022. Journal: Comput Math Methods Med.

Wu Youke's essay on epidemic disorders during the Ming Dynasty inspired Dayuan Decoction. Betel nut (6 g), Magnolia officinalis (3 g), grass nut (1.5 g), *Anemarrhena asphodeloides* (3 g), peony (3 g), *Scutellaria baicalensis* (3 g), and licorice (1.5 g)” are the ingredients in this treatment [2]. Clinical studies have shown that the Dayuan Decoction is superior to antibacterial and antiviral medications in the treatment of febrile disorders [3]. It can be used to treat various types of fever, including infectious, damp heat, persistent, high, evening, post, intermittent, and low fever [4]. It is particularly effective in the treatment of infectious and damp heat fever [5]. According to an experimental study, Dayuan decoction exhibits a substantial antipyretic effect and may help the patient cool down gently without having a high or low impact [6]. It is possible that the mechanism is to reduce excitatory stimulation to the temperature center by reducing the content of prostaglandin E2 in the cerebrospinal fluid, or by reducing serum interleukin-6 (IL-6) and tumor necrosis factor (TNF)—and myeloperoxidase activity in liver tissues, or a combination of these mechanisms [7].

Dayuan Decoction exhibits a clear antifever effect; however, its mechanism of action remains unknown and a systematic and complete investigation is required [8]. With the development of interdisciplinary research, network pharmacology (NP) has become the focus of functional component development in the future, emphasizing the interaction between multicomponent, multitarget, and multiple diseases. This is seen from the perspective of integrity and systematicity, improved efficiency, reduced development costs, and suitability for the research and development of natural products. Presently, NP has developed a series of mature data platforms, methods, and software, such as the traditional Chinese medicine system pharmacological database and analysis platform (TCMSP). The TCMSP screens traditional Chinese medicine components and determines the relationships between component target diseases; GeneCards integrates resources including genome, transcriptome, proteome, genetics, clinical, and functional information; and Stitch database predicts the interaction between drugs and proteins. For molecular interaction networks biological pathway visualization, the software platform Cytoscape is used [9]. The NP method was used in the present study to establish a database of related targets for the treatment of fever using Dayuan Decoction, construct the network relationship between target genes and pathways, and analyze the relevant pathological pathways. The focus was also on summarizing the relevant mechanism of Dayuan Decoction for the treatment of fever and exploring its potential treatment of disease.

The article "Molecular Mechanism of Dayuan Decoction in the Treatment of Fever Based on Network Pharmacology" was published in 2022. Journal: Comput Math Methods Med.

## 2. Materials and Methods

### 2.1. Screening of Main Active Components of Dayuan Decoction

The TCMSP (http://tcmspw.com/index.ph) is a systematic pharmacological database of Chinese herbal medicines that can be used to explore the relationship between drugs, targets, and diseases. The TCMSP was used, with the keywords betel nut, *Magnolia officinalis*, grass nut, *Anemarrhena aspedoloides*, peony, *Scutellaria baicalensis*, and licorice as the main seven traditional Chinese Medicine Boards of Dayuan Decoction. The screening criteria were oral bioavailability (OB) ≥ 30%, drug likeness (DL) ≥ 0.18, and half‐life (HF) ≥ 4 to screen the main active components of Dayuan decoction.

### 2.2. Collection of Drug Ingredients and Fever Gene Targets

The related target function is one of the functions of the TCMSP, which can be used to predict the action target information of the main active components of the Dayuan decision, using UniProt (https://www.uniprot.org). The database corrects and standardizes the target information of the active components to obtain the corresponding gene targets. Using the GeneCards (https://www.genecards.org/) database with “fever” as the search term, the fever-related gene targets were retrieved. Dayuan Decoction gene targets of the main active ingredients and disease-related gene targets were obtained by selecting the intersection of the Wayne diagram to obtain the common gene target, the gene target of Dayuan Decoction for the treatment of fever, loading the search results, and saving them in Excel format. This completed the collection of all human fever-related gene data.

### 2.3. Drug Component and Protein Target Interaction Analysis

Betel nut, *Magnolia officinalis*, grass nut, *Anemarrhena aspedoloides*, peony, *Scutellaria baicalensis*, and licorice were compared by importing their main active components and target information into Cytoscape 3.7.2 (http://www.cytoscape.org/). In the software, if there are more connections between a target and other targets, the target is important and is a key node. The common gene target obtained from the Wayne diagram was imported into STRING (a search tool for the retrieval of interacting genes/proteins; https://string-db.org/), the species was set as “*Homo sapiens*,” and the protein phase of common gene targets was constructed through a protein-protein interaction (PPI) network.

### 2.4. Enrichment Analysis of Gene Ontology (GO) and Kyoto Encyclopedia of Genes and Genomes (KEGG) Pathway

The database for annotation, visualization, and integrated Disco (David) is commonly used for the annotation of gene functions. Using David (https://david.ncifcrf.gov/), the species was set as “Homo sapiens,” and GO and KEGG pathway enrichment analyses were conducted. *P* < 0.01 and enriched gene counts > 5 was the cut-off value standard to further determine the molecular signaling pathway of blue Dayuan Decoction in the treatment of fever. GO analysis is composed of three aspects, namely, the biological process (BP), cellular component (CC), and molecular function (MF), to explain the essence of genes. KEGG pathway enrichment analysis is helpful to understand the signaling pathway process and function of a gene or protein in the process of the signaling pathway.

The article "Molecular Mechanism of Dayuan Decoction in the Treatment of Fever Based on Network Pharmacology" was published in 2022. Journal: Comput Math Methods Med.

### 2.5. Data Processing

All data in this study were mapped using Cytoscape version 3.7.2 software, and the significant data with *P* value < 0.01 were selected for GO enrichment and KEGG pathway analyses.

## 3. Results

### 3.1. Main Active Compounds of Dayuan Decoction

In this study, through the TCMSP, using OB ≥ 30%, DL ≥ 0.18, and HL ≥ 4 as screening criteria, 102 main active components of Dayuan Decoction were screened, including 13 from betel nut, 9 from *Magnolia officinalis*, 11 from grass nut, 6 from *Anemarrhena*, 9 aspedoloides, 9 from peony, 22 from *Scutellaria baicalensis*, and 22 licorice. After removing duplicates, a total of 89 main active components were obtained. Each active ingredient was sorted using OB value, and the top 19 active ingredients with their respective OB values are displayed in Table 1.

### 3.2. Prediction of the Target of Dayuan Decoction in the Treatment of Fever

A total of 81 therapeutic targets related to fever were identified using the GeneCards database. The intersection of the Dayuan Decoction and fever targets was determined using the Venny platform, and 50 common targets were obtained, as shown in Figure 1.

### 3.3. PPI Network Construction

Through STRING online analysis of the 50 common targets and setting parameters to remove free target proteins, a PPI core network diagram (Figure 2) was obtained. The PPI network diagram included 34 nodes and 350 edges. The network diagram was analyzed using Cytoscape 3.7.2 software. The results showed that the average node degree value of the target protein was 20.6, maximum value was 30, and minimum value was 4. There were 23 targets with higher than average degree values, of which 13 were higher than 25. These may be the key targets involved in the treatment of fever through Dayuan Decoction. Information on the key targets and degrees is presented in Table 2.

### 3.4. Target Pathway GO Enrichment Analysis

A total of 192 GO entries were obtained through screening GO enrichment analysis from the David database, including 16 cell composition, 157 biological process, and 19 molecular function entries. The results were visually analyzed using R software to obtain a bubble diagram of the GO enrichment analysis (Figures 3–5). The abscissa represents the enrichment factor, the ordinate represents the enrichment items, the size of the bubbles represents the number of enrichments, and the color of the bubbles represents the size of the *P* value. The most involved items and numbers of biological process genes were the exogenous apoptosis (14), drug response (14), and lipopolysaccharide-mediated signaling pathway (13). The items and number of genes involved in the process of cell composition were cytoplasm (22), cytosol (20), and nucleus (19). The items and the number of genes involved in molecular function processes were protein binding (30), similar protein binding (13), and protein homopolymerization activity (12).

The article "Molecular Mechanism of Dayuan Decoction in the Treatment of Fever Based on Network Pharmacology" was published in 2022. Journal: Comput Math Methods Med.

### 3.5. KEGG Pathway Enrichment Analysis

A total of 35 enrichment entries were obtained through KEGG pathway enrichment screening (*P* < 0.01), as shown in Figure 6. Among them were diseases related to tuberculosis, hepatitis B, and trypanosomiasis, as well as cancer, PI3K Akt signaling, and TNF signaling pathways. Through cluster analysis of the 35 KEGG results, eight categories were obtained, of which those with a count of more than 10 were hepatitis B (14), American trypanosomiasis (13), TNF signaling pathway (10), influenza A (10), and *Amoeba protozooses* (10).

### 3.6. Component Target Molecular Docking Results

As shown in Figure 7, the binding energy of the three core compounds with ACE2 was less than 5kj/mol, with a stable structure and high binding activity, indicating that these compounds can directly act on host human cells, improve body immunity, and block virus invasion.

### 3.7. Construction of Target Interaction Network

The obtained active compound was predicted to the target through the TCMSP database, and then, the target information was queried through DAVID, STRING, and other databases, and the drug target-metabolic pathway-active ingredient network (Figure 8) was constructed using Cytoscape software.

## 4. Discussion

Fever is defined as an increase in body temperature over the usual range as a result of pyrogen activity or other causes [10]. Exogenous heat sources, such as bacterial endotoxins, activate neutrophils, eosinophils, and the mononuclear phagocyte system in the blood, causing them to produce and release endogenous heat sources, such as ILs, TNF, and interferons (Ifs), which then cause fever through the central nervous and circulatory systems [11]. There were 189 related targets and 65 related pathways involved in the treatment of fever with Dayuan Decoction. A total of 21 specific disease-related pathways and 54 nonspecific disease-related pathways were identified. Through enrichment using GO and KEGG, results showed that the biological process involved in the treatment of fever with Dayuan Decoction focuses on the metabolic process. Among the 49 nonspecific disease-related pathways, there are 32 metabolism-related pathways, involving the metabolic pathways of drugs, exogenous substances, and a variety of amino acids, sugar, lipids, cofactors, vitamins, energy, starch, sucrose, nitrogen, and other substances [12]. Other pathways are related to immunity, internal secretion, environmental information processing, cellular processes, and the nervous system, and the number of hsa05200: Pathways in cancer-related genes were significantly higher than the number of other pathways in the 21 specific disease-related pathways, and the specific diseases included prostate cancer, pancreatic cancer, colorectal cancer, nonsmall cell lung cancer, bladder cancer, small cell lung cancer, thyroid adenocarcinoma, endometrial carcinoma, renal cell carcinoma, glioma, and melanoma [13]. There are 13 different types of malignancies, including chronic and acute myeloid leukemia. Cancerous fever may be efficiently treated through the addition and removal of Dayuan Decoction, according to clinical observation and experimentation. Huang et al. [14], for example, employed Dayuan Decoction to cure 42 instances of malignant fever in their practice.

The article "Molecular Mechanism of Dayuan Decoction in the Treatment of Fever Based on Network Pharmacology" was published in 2022. Journal: Comput Math Methods Med.

When compared to 40 instances treated with conventional medication, the curative efficacy of Dayuan Decoction was superior, and there were no negative effects reported. Wang et al. used Dayuan Decoction in the treatment of malignant fever associated with moist heat buildup, which had a positive clinical impact as well as being gentle and steady in nature, with few negative effects and excellent tolerance [15]. The network pharmacology approach was utilized to verify the efficacy of Dayuan Decoction in this investigation. In terms of the therapeutic impact of malignant fever, it is hypothesized that Dayuan Decoction has a propensity to be effective in the treatment of cancerous fever, implying that the clinical effect of Dayuan Decoction should be investigated further.

The nonspecific disease-related route includes the nervous system signaling pathway hsa04722: neurotrophin signaling pathway, which is also known as the neurotrophin signaling pathway. Neurotrophins are involved in the differentiation of nerve cells [16]. The neurotrophin family includes nerve growth factor, brain-derived neurotrophic factor, and neurotrophins 3 and 4, all of which are important for neural development as well as higher-order activities, such as learning and memory [17]. The ability to recall information is critical. Specific disorders include neurological diseases such as Alzheimer's disease and Huntington's disease [18]. Dayuan Decoction may have a therapeutic impact on neurodegenerative illnesses, which may be further enhanced through a step excavation study. The present study has some limitations. (1) If the results are used in a clinic, the implementation conditions are strict and difficult, which can be difficult to achieve in practice. (2) Animal experiments were not performed. (3) Ethical considerations for future clinical trials have not been considered in this study.

The article "Molecular Mechanism of Dayuan Decoction in the Treatment of Fever Based on Network Pharmacology" was published in 2022. Journal: Comput Math Methods Med.

Finally, the mechanism of action of Dayuan Decoction in the treatment of fever includes a range of metabolic-centered pathways, which may be activated by the simultaneous responses of multiple target complicated pathways. This research expands the body of evidence supporting the therapeutic impact of Dayuan Decoction on malignant fever and suggests that Dayuan Decoction may have the potential to cure neurodegenerative disorders in the future. The intricacy of the chemical components of traditional Chinese medicine necessitates that this research be presented only from the standpoint of facts, and several shortcomings still exist. This requires the continued enhancement of the detection strength of the LC-MS technique and metabolomics and further investigation and validation of these findings through experimental studies.

## Figures and Tables

**Figure 1:** Venny platform for Dayuan Decoction.

**Figure 2:** PPI core network diagram of common targets.

**Figure 3:** Dayuan Decoction core target point biological process (BP) bubble chart.

**Figure 4:** Dayuan Decoction core target point cellular component (CC) bubble chart.

**Figure 5:** Dayuan Decoction core target point molecular function (MF) bubble chart.

**Figure 6:** KEGG pathway enrichment.

**Figure 7:** Core compound target molecule docking result.

**Figure 8:** Active ingredient-metabolic pathway-target network diagram.

**Table 1:** Top 19 active ingredients with their OB values in the Dayuan Decoction.

Drugs	Code	Chemical structure	OB	DL	HL
Betel nut	MOL002934	NEOBAICALEIN	104.34	0.44	16.5
Licorice	MOL00456I	Sudan III	84.07	0.59	8.99
Betel nut	MOL002932	Panicolin	76.26	0.29	16.78
Betel nut	MOL012246	5,7,4-trihydroxy-8-mcthoxy flavanone	74.24	0.26	16.85
Scutellaria	MOLOOI798	ncohcspcndin_ql	71.17	0.27	15.96
Baicalensis	MOL002927	Skulkaptlavonc II	69.51	0.44	16.14
Scutellaria	MOL0029II	2,62,4′~tctrahydroxy-6′-mcthoxychalconc	69.04	0.22	21.89
Baicalensis	MOL002937	DIHYDROOROXYLIN	66.06	0.23	17.17
Licorice	MGL001820	(E)-3-(3,5-dimcthoxy-4-hydroxyb-cnzylidcne)-2-indolinonc	65.17	0.25	6.49
Magnolia officinalis	MOLOOI783	2-(9-((3-mcthyl-2-oxopcnt-3-cn-l-yl)oxy)-2-oxo-1,2,8,9-tctrahydrofuro 12,3-h|q ui nol i n-8-y 1)propan-2-y 1 acetate	64	0.57	7.67
Magnolia officinalis	MOLOOI767	Hydroxyindirubin	63.37	0.3	44.92
Magnolia officinalis	MOLOOI736	(-)-taxiiblin	60.51	0.27	14.37
Grass nut	MOL007245	3-Mcthylkcmpicrol	60.16	0.26	16.36
Grass nut	MOLOOI721	Isaindigodione	60.12	0.41	7.17
Anemarrhena	MGL000787	Fumarine	59.26	0.83	23.46
Peony	MOLOOI8I4	(E)-3-(3,5-dimcthoxy-4-hydroxy-bcnzylidcne)-2-indolinonc	57.18	0.25	10.13
Aspedoloides	MOLOOI131	phellamunn_qt	56.6	0.39	14.89
Aspedoloides	MGL000228	(2R)-7-hydroxy-5-mcthoxy-2-phcnylchroman-4-onc	55.23	0.2	17.02
Grass nut	MOLOOI793	(E)-2-[(3-indolc)cyanomcthylcne-J-3-indol!nonc	54.59	0.32	39.04

The article "Molecular Mechanism of Dayuan Decoction in the Treatment of Fever Based on Network Pharmacology" was published in 2022. Journal: Comput Math Methods Med.

**Table 2:** Key targets summary display.

Target gene	Target protein	Value
BCL2L1	Apoptosis regulatory factor bel	30
TP53	Tumor necrosis protein P53	30
Bad	Proapoptotic protein	29
CASP8	Cysteine protease	28
CASP3	Cysteine protease S	28
BAX	Apoptosis regulator BAX	27
IL-10	Interleukin 10	27
TNF	Tumor necrosis factor	26
IL-6	Interleukin 6	25
FTB	Interleukin 2	25
BCL2	Apoptosis factor 2	25
MCL1	Myeloid leukemia protein 1	25
CXCL8	Chemokine CXCL8	25

## Data Availability

All of the data in this article is actually available.
